This article has been retracted.

# A novel competitive exact approach to solve assembly line balancing problems based on lexicographic order of vectors

**DOI:** 10.1016/j.heliyon.2023.e13925

**Published:** 2023-02-23

**Authors:** Shifu Xu, Seyed Mahdi Shavarani, Mazyar Ghadiri Nejad, Bela Vizvari, Davood Toghraie

**Affiliations:** a College of Science and Technology of Ningbo University, Ningbo, Zhejiang,315300, China; b Faculty of Mechanical Engineering & Automation, Zhejiang Sci-Tech University, Hangzhou, Zhejiang, 310018, China; c Alliance Manchester Business School, University of Manchester, Manchester, UK; d Department of Industrial Engineering, Cyprus International University, 99258 Nicosia, TRNC, Turkey; e Department of Industrial Engineering, Eastern Mediterranean University, TRNC, Turkey; f Mechanical Engineering Department, Khomeinishahr Branch, Islamic Azad University, Isfahan, Iran

**Keywords:** Assembly line balancing, Exact method, Heuristics, Lexicographic order of vectors

## Abstract

The assembly line balancing problem (ALBP) is an eminent NP-hard topic that is discussed in mass production systems with low diversity. Primarily, two types of ALBPs are discussed in the literature as type I, which aims to find the minimum number of workstations for a given cycle time, and type II, which assigns some tasks to a given number of workstations such that the maximum workstation load is minimized. To solve ALBPs, various exact, heuristic, and metaheuristic methods have been proposed. However, these methods lose their efficiency when handling large-size problems. Therefore, researchers have focused on proposing heuristic and metaheuristic algorithms to solve large-size problems, especially when they deal with real-life case problems in the industry. This study aims to present a novel and competitive exact method for solving ALBP type II based on the lexicographic order of vectors for feasible solutions. To evaluate the performance of the developed method, a group of highly used standard test problems in the literature is utilized, and the results are compared and discussed in detail. The computational results in this study specify that the developed solution approach performs efficiently and yields the best global solution of all the ALB test problems, which proves the proposed method's potential and its competitive advantage.

## 1 Introduction

Assembly lines include flow-oriented manufacturing processes consisting of workstations, as productive units, to perform operations; and various tasks are added to a product sequentially at workstations [[1], [2], [3]]. Setting up an assembly lineup is a long-standing decision, which typically needs vast capital investment. Hence, it is vital to design and balance assembly lines as efficiently as possible [4,5]. Most of the literature related to assembly lines pertains to workstation load balancing. The assembly line balancing problem (ALBP) includes assigning tasks to several workstations to optimize a given objective [[6], [7], [8]]. Two main categories of ALBPs are type-I, which minimizes the number of workstations considering a known cycle time [9], and type-II, which minimizes the cycle time considering a fixed number of workstations [10]. For such kinds of ALBPs, numerous solution approaches have been provided in the literature that is classified generally into exact, heuristic, and meta-heuristic methods [11]. One of the early studies on ALBPs was performed by Salveson [12], who presented the first mathematical model to minimize the number of workstations and workloads, simultaneously. Subsequently, Helgeson and Birnie [13], introduced a heuristic solution method, called the ranked positional weight (RPW) method, for solving the ALBPs. Arcus [14], proposed the COMSOAL method wherein random solutions are generated, and the best solution is returned as the result. In the 70s and 80s, the focus of the majority of researchers was on proposing exact algorithms to deal with different types of ALBPs. The first grouping genetic method for ALBP type-II was proposed by Falkenauer and Delchambre [15], where each task depended on a set of resources. They aimed to obtain the performance of grouping genetic algorithms in large-size grouping problems like the ALBP and bin packing problems. In the 1990s, two diverse genetic algorithms have been proposed for solving ALBP type-I [16,17]. In 1997, an algorithm based on the branch & bound technique has been proposed [18]. In this method, which is the most excellent proposed exact method up to now and called SALOME, the tasks could be assigned to the workstations from both forward and backward, simultaneously. Later on, Scholl and Becker [19], discussed the inefficiency of the nature of exact methods, especially in the case of dealing with large-size problems. Thus, to solve such problems in a meaningful time and find an acceptable solution, proposing efficient methods are vital. In recent years, Davani et al. [20] studied optimizing U-shaped ALBPs by introducing just-in-time (JIT) principles of production. They considered minimizing cycle time for a fixed number of workstations and discussed the results of different test problems, using a metaheuristic algorithm. They found that the U-shaped assembly line has a better performance considering the JIT principles. Mirzaei et al. [21] studied a real case problem of ALB at a metal manufacturing company, concerning the efficiency and smoothness indexes of the assembly line. They considered two main types of assembly lines such as type I and type II, and utilized an evolution strategy algorithm to optimize them. Moreover, utilizing a discrete-events simulation analysis, they evaluated the assembly line behavior based on the dynamic model, using a stochastic approach. The focus of the research in this area has been on proposing metaheuristic methods and competitive algorithms like evolution strategies and ANNs, grouping evolution strategies, particle swarm optimization, honey bee optimization, genetic algorithms, beam search algorithm, differential evolution approach, ant colony algorithm, and local search algorithm, in the recent decade [10,[22], [23], [24], [25], [26], [27], [28], [29], [30], [31]]. In addition to the mentioned literature, several exact methods like the branch & bound [32], linear programming [33], dynamic programming [34], integer programming [35], and mixed-integer programming [36], were proposed to solve different types of ALBPs. Recently, Fleszar [37] developed a mixed-integer linear programming (MILP) model for two different ALBPs. In the first one, each task contains only one compatible workstation; in the other one, each task can be compatible with multiple workstations. These models could find 81% of the optimal solutions from 1200 problem instances. Subsequently, Bora et al. [38] studied a robotic ALBP in which the task time depends on the robot assigned to each station. Considering the branch & bound method, they proposed a mixed integer model, and a heuristic solution method to solve problem. A significant disadvantage of exact methods is that they are time-consuming especially when the number of operations and workstations increases. To define the lexicographic order method, it should be noted that the assembly line balancing has two types of problems as two main objective functions are relevant to it. Even further objective functions can be introduced. A sequence of papers used a multi-objective function approach. They applied a method of goal programming such that the objective functions are in a strict order [[39], [40], [41], [42], [43], [44], [45]]. In such methods, the procedure is to optimize the first objective function initially. If an optimal solution is reached, then a new constraint is created by restricting the first objective function on that value. Then, a new problem is developed to improve the other objective function. If the optimality is reached, then the value of this objective function is also fixed. The third objective function is optimized in the third problem, and so on. This strict order of the objective functions is called the multi-objective decision-making lexicographic order. Primarily, Sawik proposed a bi-objective integer formulation to optimize a flexible assembly line. He developed a new heuristic solution method when both the loadings and routing problems have been considered in the system, simultaneously [46]. Pastor introduced the lexicographic bottleneck ALBP for not only minimizing the highest workload when the number of the workstations is known and fixed but even for obtaining a smooth assignment of the tasks [47]. This approach has m-1 objective functions, where m is the number of workstations. The word “lexicographic” concerns the above-mentioned order of the objective function. He developed two mixed-integer linear programming to solve the problem. Pastor et al. [48], proposed a new heuristic method to solve the mentioned lexicographic bottleneck ALBP by using the local search algorithm, where the initial solution was generated by another heuristic procedure. In recent years, Kucukkoc et al. [49] proposed an artificial bee colony method for the lexicographic bottleneck mixed-model ALBP. Considering the mentioned lexicographic methods, in this study, the potentially feasible solutions are enumerated in the lexicographic order, which is different from the approach utilized in the mentioned studies. In the mentioned above studies the order is considered for the objective functions but in the present study, the order is applied for the potentially feasible solutions that are enumerated. Here, the only objective function is the cycle time. The potentially feasible solutions of the assignments to the workstations are ordered lexicographically. Using such a modification, the proposed approach in this study is a lexicographic order-based algorithmic tool for obtaining fast and exact enumeration to solve ALBP type-II. This method is an enumeration method that uses a cutting point to prohibit the search within the infeasible region, and consequently reduces the solution space and CPU time significantly, where the assignment of each station is described by a binary vector. Distinguished standard test problems, found in the literature, are utilized to evaluate the performance of the proposed method in this study. The content of this study is the following: In the next section, the problem definition and assumptions are described. Section 3 includes the developed solution method. The computational and obtained results are covered in section 4. The comparative analysis is done in the fifth section, and finally, the study is concluded in the last section.

## 2 Problem definition

To minimize the cycle time of single-product manufacturing with a known fixed number of workstations, ALBP type-II, the necessary assumptions, and definitions are listed as follows:

- The precedence diagram, containing all the predecessors and successors of tasks, is given.
- All tasks are accessible in the beginning.
- The processing times of tasks are fixed. The processing time of task *i* is *ti* time unit.
- Tasks may not be divided into two or more workstations, and each task should be assigned to one and only one station. In other words, each task must be processed and completed in only one workstation.
- Allocation limitation is non-existent except for precedence limitations.
- A task can be processed in any workstation given that its predecessors are processed in the previous or at the same workstation.

Nomenclature

ISet of existing tasks ($i,i^{\prime }\in I$)
JSet of workstations ($j,j^{\prime }\in J$)
mTotal number of workstations
$x_{ij}=\left\{ \begin{array}{cc} 1 & if\;task\;i\;is\;assigned\;to\;workstation\;j\;\\ 0 & otherwise\; \end{array}\right.$

$${Pre}_{i^{\prime }i}=\left\{ \begin{array}{cc} 1 & if\;taski^{\prime }\;is\;immediate\;predecessor\;of\;task\;i\;\\ 0 & otherwise\; \end{array}\right.$$

$$t_{i}=Processing\;time\;of\;task\;i$$

C: Cycle time

Various mathematical formulations have been presented to solve diverse types of ALBPs in the literature, e.g., the first one that was developed by Bowman [50]. In the following, one of the recent mathematical models for solving ALBP type-II, prepared by Zheng et al. [51] is presented.

(1) minimizeC

Subject to:

(2) $$\sum_{j=1}^{m}x_{ij}=1\forall i=1,\ldots ,n$$

(3) $$\sum_{j=1}^{m}{jx}_{ij}\leq \sum_{j^{\prime }=1}^{m}{j^{\prime }x}_{i^{\prime }j^{\prime }}\forall i,i^{\prime }=1,\ldots ,n\;{|}_{{Pre}_{ii^{\prime }}=1}$$

(4) $$\sum_{i=1}^{n}{t_{i}x}_{ij}\leq C\forall j=1,\ldots ,m$$

(5) $$x_{ij}=0,1\forall i=1,\ldots ,n,j=1,\ldots ,m$$

In the mentioned mathematical formulation, the objective function is defined by equation (1), which is related to minimizing the cycle time. Constraint (2), force each task to be assigned to one and only one workstation, where *n* tasks and *m* workstations exist. Constraint (3) ensures that the precedence conditions are considered. Inequality (4) implies that the access time for every workstation may not be more than the cycle time, and finally, constraint (5) defines all the decision variables of *x*_*ij*_ as binary variables.

## 3 Solution method

The procedure of the proposed method in this study contains three steps. First, the traditional lexicographic order of vectors should be introduced. In the second step, the order is discussed in the Boolean case, *i.e*., 0–1 vectors, and finally, it is used to obtain an implicit enumeration scheme for assigning the tasks to the workstations.

### 3.1 The lexicographic order of vectors

To explain the lexicographic order of vectors, initially, it should be defined that the order of objects is a partial order if incomparable pairs of objects exist. Additionally, a well-known partial order is the component-wise order of vectors. The vectors $u,w\in R^{2}$ are incomparable if they contain a pair of components with opposite magnitudes. For example, $u_{1}<w_{1}$ and $u_{2}>w_{2}$ or the opposite, *i.e*., $u_{1}>w_{1}$ and $u_{2}<w_{2}$. The lexicographic order is complete as any two vectors having the same dimension are comparable, because it follows immediately from the definition of the lexicographic order.

Definition 3.1 Let $u,w\in R^{n}$ be two n-dimensional vectors. The vector u is lexicographically smaller than the vector w if an index k(1≤k≤n) exists such that a) $u_{i}=w_{i}\;i=1,\ldots ,k-1$, and b) $u_{k}<w_{k}$. This relation is denoted by u ◄w.

Every order is determined by a cone in linear spaces. The relation u ◄w is true if and only if a vector v exists such that u+v=w, and

$$v\in \left\{t\in R^{n}:t_{1}>0\right\}\cup \left\{t\in R^{n}:t_{1}=0,t_{2}>0\right\}\cup \ldots \cup \left\{t\in R^{n}:t_{i}=0,i=1,\ldots ,n-1,t_{n}>0\right\}\text{.}$$

### 3.2 The lexicographic order in the case of Boolean vectors in a general and a constrained problem

Lexicographically, the greatest vector is (1,1, …,1,1), and the second greatest vector is (1,1, …,1,0). Let's assume that u is a non-zero binary vector, as only finite Boolean vectors exist. Subsequently, an index t may exist such that $u_{t}=1,u_{t+1}=\ldots =u_{n}=0\text{.}$ In the lexicographical decreasing order, the next vector is v with $u_{i}=v_{i}\;\left(i=1,\ldots ,t-1\right),v_{t}=0,v_{t+1}=1,\ldots ,v_{n}=1\text{.}$ Consequently, the zero vector is the lexicographically minimal binary vector, and no vector exists thereafter. In the method described below, binary vectors are used to identify the tasks assigned to the workstations. Each workstation has its binary vector like $u^{j}$ such that it is component $u_{i}^{j}$ is 1 if operation i is assigned to workstation j and 0, otherwise. Assume that a feasible vector exists such as u, where $u_{1}=\ldots =u_{t}=1,u_{t+1}=\ldots =u_{n}=0$. Subsequently, the vector v is feasible such that $v_{i}=u_{i}\;\left(i=1,\ldots ,t-1\right),v_{t}=v_{t+1}=\ldots =v_{n}=0$. Therefore, the next lexicographical feasible vector is generated using Eqs. (6), (7), (8).

(6) v(t)=v

(7) $${v\left(k\right)}_{i}={v\left(k-1\right)}_{i}\;i=1,\ldots ,k-1,k+1,\ldots ,n;\forall k=t+1,\ldots ,n$$

(8) $${v\left(k\right)}_{k}=\begin{array}{cc} 1 & if\;v\left(k\right)+e_{k}\;is\;feasible\\ 0 & if\;v\left(k\right)+e_{k}\;is\;not\;feasible \end{array}$$

where $e_{k}$ is the $k^{th}$ unit vector.

The ALBP comprises two types of constraints including that a load of a workstation may not exceed the cycle time, and the assigned tasks must satisfy the precedence relation. Both constraints exhibit the following properties:

(a) If a set of tasks satisfies the constraints, then all of its subsets satisfy the constraints as well.
(b) If a set (S) of tasks violates the constraints, then all sets T violate the constraints as well if S⊂T. This property enables many infeasible orders to be skipped and larger steps to be performed in the lexicographical enumeration of the binary vectors. The key point is that the enumeration leaps from one feasible vector to the next feasible vector, lexicographically. The proposed algorithm starts with the calculation of the upper and lower bounds of the cycle time that are calculated by equation (9).

(9) $$\mathrm{Max}\left(\frac{\alpha \sum_{i=1}^{n}t_{i}}{m},{\alpha t}_{i}\right)$$

where α is an arbitrary coefficient such that α>1. A large value for α would increase the CPU time, and a small value would increase the risk of losing the feasibility. In this study, and after some initial experiments, α is considered equal to 1.5. The lower bound is calculated by equation (9), considering α=1. The upper bound is used as the initial value for the cycle time and the lower bound is considered as the stopping criteria. It should be mentioned that in case of obtaining a non-integer value for the upper bound, the value is rounded up. To initiate the algorithm, tasks are first ordered based on the total number of successive tasks. The higher the total number of successive tasks, the lower the order of the task; and consequently, the higher the priority of its assignment. In the case of ties, priority is given to the task with a higher processing time. The algorithm starts with assigning the first activity to the first station and continues assigning subsequent tasks individually according to their order to the same workstation while the load of the workstation does not exceed the cycle time; subsequently, it proceeds to the next workstation. The algorithm continues until all the tasks are assigned to the workstations. It is obvious that the ending task, *i.e*., a task with no successor is always assigned to the last workstation if only one task exists. If more than one starting task exists, a dummy task is added before them, to serve as the starting task by setting all the original starting tasks as the successors of this dummy task. Similarly, if more than one ending task exists, a dummy task is considered to serve as the ending task, and the original ending task will be its predecessor. If a feasible solution is found, then C becomes less than the best cycle time by a one-time unit. The algorithm verifies the first workstation to confirm whether the assigned load has violated the cycle time. If the cycle time is not violated, the next workstation is evaluated; however, if the cycle time is violated, the assignment vector of the workstation is changed to the next lexicographic order. The assignment vector would change continuously to the next lexicographic order until the load of the workstation is less than the cycle time and the assignment is feasible. If a zero vector is reached, the algorithm would return to the previous workstation and attempt to obtain the next feasible lexicographic order for that station. To avoid complete enumeration, a cutting criterion is considered whenever the assignment of tasks to a workstation is completed. When the assignment of the $i^{th}$ workstation is completed, the algorithm would verify the feasibility of the incomplete solution to avoid the complete enumeration of the feasible area. The partial solution is infeasible if equation (10) is not violated.

(10) $$\frac{\sum_{i+1}^{n}t_{i}}{m-i}>C$$

In this case, the next lexicographic order of the assignment vector is considered for the $i^{th}$ workstation until the feasibility of the partial solution is satisfied. At the end of each iteration, the successful assignment and the corresponding cycle time are saved as the best solution found, and the algorithm continues to the next iteration by reducing the value of C, with one unit, and beginning the procedure from the first workstation. The algorithm stops if no feasible solution is found for the updated C, and the best-recorded solution in the previous iteration is returned by the algorithm. In the proposed algorithm, two important points are noteworthy. The first one is that obtaining the next feasible lexicographic order of an assignment vector for a workstation may lead to a zero vector. In this case, the lexicographic order change would proceed to the previous workstation. The second point is while attempting to determine the assignment of a specific workstation, the proceeding workstation is considered unassigned, implying that zero vectors exist for the next workstations. The assignment is performed only for those tasks that have not been assigned to the previous workstations. The algorithm returns to the previous workstation if the assignment vector changes to zero vector during the change to the next feasible load on the lexicographic order. If this chain of changes returns to the first workstation and it changes to a zero vector, no feasible solution for the specified cycle time is implied, and the algorithm stops at this point. The pseudocode of the algorithm is illustrated in Fig. 1.

**Table:** 

Rank the tasks based on the total number of successors
Calculate Upper and Lower bounds
C ← upper bound
Assign tasks to each workstation such that for each workstation j we have $\sum_{j}t_{i}x_{ij}\leq C$
Best ←C
While C≥Lowerbound
C = C – 1
For workstation i=1:m−1
While $\sum_{j}t_{i}x_{ij}\geq C$ and if $\frac{\sum_{i+1}^{n}t_{i}}{m-i}>C$
Change the assignment vector to the next lexicographic order
If the assignment vector is zero vector
If i=1
finish the algorithm and return the Best
Else
i←i−1
End If
End If
End While
End For
Best = C
End while
Return Best

**Fig. 1:** Pseudocode of the lexicographic algorithm.

The flowchart of the proposed lexicographic algorithm has been illustrated in Fig. 2.

**Fig. 2:** Flowchart of the proposed Lexicographic algorithm.

To explain how the proposed algorithm solves the ALBPs based on the proposed lexicographic method in this study, a precedence diagram comprising 12 tasks, to be assigned to 3 workstations, m = 3, is considered [22]. Fig. 3 illustrates the predecessors and successors of each task and the task times that are mentioned at the top of each node.

**Fig. 3:** Sample of the precedence graph.

According to the precedence graph, Fig. 3, the first task is assigned to workstation 1 first. Then, one task among tasks 2 and 4 is chosen to be assigned to workstation 1 or workstation 2, if the idle time of the first workstation is insufficient. Similarly, the other task is assigned to the workstations up to assigning all the tasks. The proposed algorithm is as follows:

Step 1 Calculate the number of total successors for each task. Table 1 shows the number of successors for each task in the precedence graph shown in Fig. 3.

**Table 1:** The total number of successors for the activities is given in Fig. 3.

Task no.	1	2	3	4	5	6	7	8	9	10	11	12
Total successors numbers	11	8	7	8	7	6	2	1	1	2	1	0

Step 2 Order the activities based on the total number of successor activities obtained in step 1. In the case of ties, the activity with a greater task time is selected; in case the task times are also equal, one of them is selected randomly. Table 2 presents the order of the tasks and their corresponding number of successors in decreasing order.

**Table 2:** Order of the activities based on step 2.

Task no.	1	2	4	5	3	6	10	7	8	11	9	12
Total number of successors	11	8	8	7	7	6	2	2	1	1	1	0

Step 3 The upper and lower bounds of the cycle time are calculated using equation (9). The obtained lower bound is equal to 17 considering α=1 and m=3. The upper bound is equal to 25.5 considering α=1.5 using similar calculations. After rounding up, the upper bound will be 26-time units.

Step 4 The initial assignment is performed as explained before, and its results are as shown in Table 3, by considering a cycle time of 26:

**Table 3:** Instant problem - initial assignment.

Task no.	1	2	4	5	3	6	10	7	8	11	9	12	Load
Task Processing Time	5	3	3	6	4	5	4	2	7	4	1	7	
Workstation 1	1	1	1	1	1	1	0	0	0	0	0	0	26
Workstation 2	0	0	0	0	0	0	1	1	1	1	1	1	25
Workstation 3	0	0	0	0	0	0	0	0	0	0	0	0	0

Step 5 Considering the initial solution, which is acquired in step 4, and the cycle time which is equal to 26, the next iteration starts by considering the cycle time = 26–1 = 25. It is obvious that the load of the first workstation exceeds that of the cycle time; thus, the next lexicographic order of the assignment vector is considered. Furthermore, all the assignment vectors for the workstations after the current workstation are set equal to zero. If the next lexicographic order satisfies the feasibility conditions, the assignment continues to the last workstation, as explained. Therefore, the results of the next iteration are as shown in Table 4.

**Table 4:** Instant problem - second iteration.

Task no.	1	2	4	5	3	6	10	7	8	11	9	12	Load
Task Processing Time	5	3	3	6	4	5	4	2	7	4	1	7	
Workstation 1	1	1	1	1	1	0	0	0	0	0	0	0	21
Workstation 2	0	0	0	0	0	1	1	1	1	1	1	0	23
Workstation 3	0	0	0	0	0	0	0	0	0	0	0	1	7

The cycle time here is 23; this solution is saved as the best solution and the next iteration starts with a cycle time of 22; the results are illustrated in Table 5.

**Table 5:** Instant problem - third iteration.

Task no.	1	2	4	5	3	6	10	7	8	11	9	12	Load
Task Processing Time	5	3	3	6	4	5	4	2	7	4	1	7	
Workstation 1	1	1	1	1	1	0	0	0	0	0	0	0	21
Workstation 2	0	0	0	0	0	1	1	1	1	1	0	0	22
Workstation 3	0	0	0	0	0	0	0	0	0	0	1	1	8

At the end of the previous step, the cycle time is 22, therefore the cycle time of 21 is considered for the next step the results are shown in Table 6. Additionally, the algorithm would continue until the stopping criteria are fulfilled. Table 7, Table 8, Table 9, illustrate the results of the repetition of performing similar steps, especially the change in assignment vectors into the next lexicographic.

**Table 6:** Instant problem - fourth iteration.

Task no.	1	2	4	5	3	6	10	7	8	11	9	12	Load
Task Processing Time	5	3	3	6	4	5	4	2	7	4	1	7	
Workstation 1	1	1	1	1	0	0	0	0	0	0	0	0	17
Workstation 2	0	0	0	0	1	1	1	1	0	1	1	0	20
Workstation 3	0	0	0	0	0	0	0	0	1	0	0	1	14

**Table 7:** Instant problem - fifth iteration.

Task no.	1	2	4	5	3	6	10	7	8	11	9	12	Load
Task Processing Time	5	3	3	6	4	5	4	2	7	4	1	7	
Workstation 1	1	1	1	1	0	0	0	0	0	0	0	0	17
Workstation 2	0	0	0	0	1	1	1	1	0	1	0	0	19
Workstation 3	0	0	0	0	0	0	0	0	1	0	1	1	15

**Table 8:** Instant problem - sixth iteration.

Task no.	1	2	4	5	3	6	10	7	8	11	9	12	Load
Task Processing Time	5	3	3	6	4	5	4	2	7	4	1	7	
Workstation 1	1	1	1	1	0	0	0	0	0	0	0	0	17
Workstation 2	0	0	0	0	1	1	1	1	0	0	1	0	16
Workstation 3	0	0	0	0	0	0	0	0	1	1	0	1	18

**Table 9:** Instant problem - last iteration; optimal results achieved.

Task no.	1	2	4	5	3	6	10	7	8	11	9	12	Load
Task Processing Time	5	3	3	6	4	5	4	2	7	4	1	7	
Workstation 1	1	1	1	1	0	0	0	0	0	0	0	0	17
Workstation 2	0	0	0	0	1	1	1	0	0	1	0	0	17
Workstation 3	0	0	0	0	0	0	0	1	1	0	1	1	17

As the cycle time is 17, which is equal to the lower bound of the problem, the algorithm is stopped.

## 4 Results and discussions

In this part, outputs obtained by applying the proposed method for various standard ALB test problems are presented and compared to the best-found solutions in the literature [18]. 16 different test problems have been considered in the literature, which can be also found in the “www.assembly-line-balancing.de” website address. To solve these problems, the proposed method has been coded in MATLAB R2016b, and a computer with Intel(*R*) Core(*TM*) *i*5-3320 M CPU@ 2.60 GHz and 4.00 GB of RAM properties were utilized. Table 10 shows the names and details of the used standard test problems.

**Table 10:** Characteristics of the test problems.

Problem no.	Name	Task no.	t_min_	t_max_	t_sum_	Station no. (min-max)
1	Arcus1	83	233	3691	75707	3–7
2	Arcus2	111	10	5689	150399	3–13
3	Barthold	148	3	383	5634	3–15
4	Barthol2	148	1	83	4234	27–33
5	Buxey	29	1	25	324	7–14
6	Gunther	35	1	40	483	6–15
7	Hahn	53	40	1775	14026	3–6
8	Kilbridge	45	3	55	552	3–11
9	Lutz1	32	100	1400	14140	8–12
10	Lutz2	89	1	10	485	9–24
11	Lutz3	89	1	74	1644	3–6
12	Mukherje	94	8	171	4208	3–15
13	Sawyer	30	1	25	324	7–14
14	Tonge	70	1	156	3510	3–20
15	Warnecke	58	7	53	1548	3–20
16	Wee-Mag	75	2	27	1499	3–11

In Table 10, the first two columns from the left, are related to the test problem numbers and the test problem names. The third column entitled “*Task no.*”*,* contains the number of activities in the related test problem. In the next three columns, *t*_min_ is the least task time among all the tasks, *t*_max_ is the supreme task time among all tasks, and *t*_*sum*_ is the summation of all the task times of the related test problem. Finally, the last column entitled “*Station no. (min-max)*” illustrates the given minimum and the maximum number of workstations used to test the proposed method. For instance, in the first row of Table 10, the test problem of Arcus1, which has been solved considering 3 to 7 workstations has been shown. Table 11 presents the results of solving the test problems mentioned in Table 10. In this table, the first column shows the name of the test problems. The second column is related to the number of tasks in each of the test problems. Columns 3 to 5 indicate the number of workstations, minimum cycle time, and CPU time for solving the test problems, respectively. Since the proposed method in this study yields the optimal solution for all of the test problems, only one column is related to the optimal solution, and the results of the proposed method are in Table 11. The optimal results are consistent with those found using the SALOME method [18].

**Table 11:** Computational results.

Problem Name	Task no.	Station no.	CT_min_	CPU time	Problem Name	Task no.	Station no.	CT_min_	CPU time
Arcus1	83	3	25236	0.050018	Barthold	148	3	1878	0.026087
		4	18927	0.027358			4	1409	0.003932
		5	15142	0.013023			5	1127	0.004714
		6	12620	10.97206			6	939	0.005482
		7	10826	5259.247			7	805	0.007649
Arcus2	111	3	50133	0.030833			8	705	0.006914
		4	37600	0.051592			9	626	0.00717
		5	30080	4.342124			10	564	0.007937
		6	25067	5.038344			11	513	0.006933
		7	21486	0.09431			12	470	0.007828
		8	18800	1900			13	434	0.010846
		9	16711	4813			14	403	0.00856
		10	15040	26177.51			15	383	0.009722
		11	13673	21339.25	Barthol2	148	27	157	0.047953
		12	12534	1043.52			28	152	0.053102
		13	11570	21875.44			29	146	0.040982
Buxey	29	7	47	0.00721			30	142	0.040913
		8	41	0.011969			31	137	0.039101
		9	37	0.01176			32	133	0.052415
		10	34	0.014461			33	129	0.133663
		11	32	0.214504	Gunther	35	6	84	0.040712
		12	28	0.048124			7	72	0.265287
		13	27	0.333213			8	63	0.106913
		14	25	0.002473			9	54	0.004255
Hahn	53	3	4787	5.36127			10	50	0.784014
		4	3677	10.84475			11	48	79.89677
		5	2823	9.388964			12	44	49.71911
		6	2400	9.711796			13	42	19.63893
Lutz1	32	8	1860	1.489377			14	40	3.490969
		9	1638	1.283405			15	40	0.004175
		10	1526	21.44104	Kilbridge	45	3	184	0.002088
		11	1400	0.021154			4	138	0.002647
		12	1400	0.003758			5	111	0.003653
Lutz2	89	9	54	0.013565			6	92	0.002424
		10	49	6704.323			7	79	0.003726
		11	45	0.008059			8	69	0.003703
		12	41	0.008155			9	62	0.002624
		13	38	0.008911			10	56	0.003023
		14	35	0.008413			11	55	0.003121
		15	33	0.009132	Mukherje	94	3	1403	0.014112
		16	31	0.007148			4	1052	0.003938
		17	29	0.386422			5	844	0.107466
		18	28	0.047073			6	704	0.076401
		19	26	0.016474			7	621	0.790043
		20	25	0.014592			8	532	0.213572
		21	24	0.013449			9	471	0.151683
		22	23	0.008262			10	424	0.16644
		23	22	0.054728			11	391	0.388565
		24	21	0.44395			12	358	0.376609
Lutz3	89	3	548	0.021319			13	325	0.060579
		4	411	0.004997			14	311	0.651948
		5	329	0.002754			15	288	0.464285
		6	275	0.278935	Tonge	70	3	1170	0.004253
Sawyer	30	7	47	0.028643			4	878	0.0029
		8	41	0.002853			5	702	0.011618
		9	37	0.016566			6	585	0.034986
		10	34	0.042451			7	502	0.013562
		11	31	0.029749			8	439	0.052776
		12	28	0.074986			9	391	3.212833
		13	26	0.010474			10	352	5.791914
		14	25	0.003686			11	320	0.016679
Warnecke	58	3	516	0.015724			12	294	148.5435
		4	387	0.00458			13	271	0.733759
		5	310	0.002747			14	251	9.937133
		6	258	0.006073			15	235	589.2252
		7	222	0.004299			16	221	200.4705
		8	194	0.0059			17	208	301.8382
		9	172	0.055541			18	196	0.782658
		10	155	0.079969			19	186	307.9366
		11	142	0.19243			20	177	121.1767
		12	130	0.165852	Wee-Mag	75	3	500	0.011823
		13	120	0.060187			4	375	0.004314
		14	111	0.010754			5	300	0.003259
		15	104	0.209831			6	250	0.002401
		16	98	0.128625			7	215	0.008197
		17	92	0.486241			8	188	0.005199
		18	87	0.109184			9	167	0.003066
		19	84	36.29672			10	150	0.024964
		20	79	12.04962			11	137	0.007398

As shown from the results in Table 10, 146 out of 158 problems have been solved in less than 3 min using the proposed lexicographic method. Four test problems have been solved between 3 and 10 min, and only eight test problems have been solved in more than 10 min. From another perspective, all the test problems related to Bartold, Bartol2, Buxey, Gunter, Hahn, Kilbridge, Lutz1, Lutz 3, Mukherje, Sawyer, Tonge, Warnecke, and Wee-Mag, have been solved in less than 10 min that shows the efficiency of the proposed lexicographic method.

## 5 Comparative analysis

To analyze the efficiency of the proposed method in this study, the results of the grouping evolution strategy method (GES) have been considered. GES is one of the efficient methods to solve ALBPs according to the literature. Different standard test problems are considered to compare the proposed lexicographic method in this study and the GES method, according to Table 12. The name of the test problems, task times, cycle time, obtained workstation numbers, and the CPU time for the GES method have been listed in Table 12. Additionally, the results obtained by the proposed lexicographic method have been listed in the last two columns of the table. According to Nejad and Kashan [], to solve these problems using the GES method, a computer with Intel(*R*) Core(*TM*) *i*5-3470 CPU@ 3.20 GHz and 8.00 GB of RAM properties have been utilized, and the method has been coded in MATLAB R2017a. It is seen that the utilized technology in their research, has significantly higher performance than the utilized software and computer in this study.

**Table 12:** Comparative results between the GES and the proposed Lexicographic method.

Problem name	Task no.	GES			Lexicographic	
		Cycle Time	Obtained Workstations	CPU time (Sec)	Optimal Workstations	CPU time (Sec)
Buxey	29	33	11	14.82	11	0.214504
		41	9	11.856	8	0.011969
		54	7	10.826	7	0.00721
Gunther	35	41	14	21.075	14	3.490969
		54	10	14.578	9	0.004225
		81	7	12.48	7	0.2265287
Hahn	53	2806	6	13.431	6	9.711796
		4676	4	12.105	4	10.84475
Lutz1	32	1414	11	14.976	11	0.021154
		1768	9	13.353	9	1.283405

The results in Table 12 show that among 10 test problems, 8 optimal answers have been obtained by the GES algorithm but all of the optimal answers have been obtained by the proposed Lexicographic method. Additionally, the average CPU time for the GES algorithm is 13.95 s while the average time of the Lexicographic method is 2.58 s. The results illustrate that the proposed Lexicographic method is significantly more efficient than the GES method.

## 6 Conclusion

In this study, a general ALBP, considering minimization of the cycle time, given several workstations, ALBPs type-II, was considered. To solve such a problem, a novel exact method based on the lexicographic order of vectors was presented. Using well-known test problems in the literature, the proposed method was solved and the results were compared to the obtained optimal answers by the SALOME method proposed by Scholl and Klein [18]. The experimental results and the performance of the proposed lexicographic method illustrated that the optimal global solutions of all ALBP test problems were obtained, efficiently. Moreover, the obtained results were compared to the results of the grouping evolution strategy (GES) method presented by Nejad and Kashan []. This method is one of the recent metaheuristic methods and one of the most efficient ones among the presented algorithms in the literature, especially for solving straight-line layouts of ALBPs. The evaluations proved that the CPU time of the proposed method is significantly less that the GES metaheuristic algorithm. Additionally, the GES algorithm cannot obtain the global optimal solutions for all of the test problems. As the proposed lexicographic-based method was so effective for solving ALBPs type-II, the authors are adapting a similar lexicographic solution approach for solving ALBPs type-I, which is the minimization of the number of workstations, given the value of the cycle time. Moreover, the method proposed in this study has enough potential to be adjusted for solving traditional scheduling and optimization problems such as bin packing, knapsack, set covering problems, etc. that can be considered as future studies.

## Author contribution statement

Shifu Xu; Seyed Mahdi Shavarani: Conceived and designed the experiments; Analyzed and interpreted the data; Contributed reagents, materials, analysis tools or data; Wrote the paper.

Mazyar Ghadiri Nejad: Conceived and designed the experiments; Performed the experiments; Analyzed and interpreted the data; Contributed reagents, materials, analysis tools or data; Wrote the paper.

Bela Vizvari; Davood toghraie: Performed the experiments; Analyzed and interpreted the data; Contributed reagents, materials, analysis tools or data; Wrote the paper.

## Funding statement

This work was supported by the General Project of Education Department of Zhejiang Province (Y201737089), Project of Educational Science Planning in Zhejiang Province (2022SCG111), National Innovation and Entrepreneurship Program for College Students (202113277010, 202213277003) and University-level Scientific Research Fund (XYL20016, YK202208).

## Data availability statement

No data was used for the research described in the article.

## Declaration of interest’s statement

The authors declare no competing interests.
